RETRACTED

# Intelligent Advisory Speed Limit Dedication in Highway Using VANET

**DOI:** 10.1155/2014/629412

**Published:** 2014-06-04

**Authors:** Ali Jalooli, Erfan Shaghaghi, Mohammad Reza Jabbarpour, Rafidah Md Noor, Hwasoo Yeo, Jason J. Jung

**Affiliations:** ^1^Department of Computer System and Technology, University of Malaya, 50603 Kuala Lumpur, Malaysia; ^2^Department of Civil and Environmental Engineering, Korea Advanced Institute of Science and Technology, Daejeon 305701, Republic of Korea; ^3^Department of Computer Engineering, Yeungnam University, Gyeongsan 712749, Republic of Korea

## Abstract

Variable speed limits (VSLs) as a mean for enhancing road traffic safety are studied for decades to modify the speed limit based on the prevailing road circumstances. In this study the pros and cons of VSL systems and their effects on traffic controlling efficiency are summarized. Despite the potential effectiveness of utilizing VSLs, we have witnessed that the effectiveness of this system is impacted by factors such as VSL control strategy used and the level of driver compliance. Hence, the proposed approach called Intelligent Advisory Speed Limit Dedication (IASLD) as the novel VSL control strategy which considers the driver compliance aims to improve the traffic flow and occupancy of vehicles in addition to amelioration of vehicle's travel times. The IASLD provides the advisory speed limit for each vehicle exclusively based on the vehicle's characteristics including the vehicle type, size, and safety capabilities as well as traffic and weather conditions. The proposed approach takes advantage of vehicular ad hoc network (VANET) to accelerate its performance, in the way that simulation results demonstrate the reduction of incident detection time up to 31.2% in comparison with traditional VSL strategy. The simulation results similarly indicate the improvement of traffic flow efficiency, occupancy, and travel time in different conditions.

## 1. Introduction

Traffic safety professionals continue to be concerned regarding heavy casualties which are taking place in highways, owing to lack of drivers' knowledge about the current safe speeds. Despite reduction in the overall numbers of speed-related crashes and fatalities, the ratio of speed-related fatalities on highways has remained unchanged about one-third of crashes and fatalities over the last quarter century [1]. As this factor is a main determinant of crash severity, it should not be any surprise that high percentage of highway deaths involves speeding [2]. Moreover, the consideration of speed safety has an essential role in increasing the road safety for the reason that, in addition to affecting the severity of crashes, it is associated with the risk of being involved in a crash [3]. Relationship between speed and crash rate is deeply discussed by several authors [3–5]. By going through consideration of safe speed as a significant factor for improving the traffic efficiency and safety, various criteria evolve which affect the procedure of decision making about the safe speed along the highways. The two most remarkable criteria comprise (1) adverse weather conditions (e.g., rain, snow, fog, etc.) which increases the number of vehicle crashes due to reduction of visibility, vehicle stability, and maneuverability; (2) traffic states such as sudden congestions, which lead to shockwave propagations and increase the probability of accident occurrence [5]. Therefore, to minimize the road hazards, drivers should be informed about the road conditions so that the drivers can adjust their speed according to the road conditions as long as they are warned about congested road conditions.

RETRACTED

VSLs are designed to improve traffic flow fluency, enhance road safety by reducing speed difference, and decrease CP in specific locations of highways which have critical potential of congestion. Unlike traditional static speed signs, VSL system allows roadway system managers to display a maximum speed limit based on current conditions which have effect on roadway performance. For instance, in case of unpredicted traffic congestion occurrence, the amount of required deceleration for upstream vehicles in free flow increases rear-end collision likelihood; hence providing sufficient space for upstream high speed vehicles is necessity before they encounter a traffic queue. The VSLs have been studied for decades to present most efficient technique to inform drivers about operating their vehicles in a way that enhances road safety [6]. Despite the potential effectiveness of utilizing VSL for enhancing road safety and traffic flow efficiency, the utilization of current VSLs for improving the traffic controlling in highways has constantly been involved with expense of increasing the average travel time of vehicles up to 23 percent [7]. Hence, reduction of average travel time has always been a challenge that different VSL strategies have confronted with. In addition, the lack of driver compliance to the advisory speed limits owing to absence of differentiation between different types of vehicles leads to decreasing the efficiency of VSL systems.

Nowadays by evolving the new intelligent technologies as an impressive contributor of transportation systems, the employing of ITS [8] concept has greatly reaped attention of governments and academia in this area. Meanwhile, the use of VANET as a subset of MANET is the significant wireless technology proposed exclusively for vehicular environment using the WAVE spectrum. The utilization of this technology in ITS is the concept which is prominently demonstrated to enhance the road safety, efficiency, and services [9] through real-time V2V and V2I communications. Accordingly, this paper attempts to address the aforementioned deficiencies of current VSL systems by taking advantage of speed limit information dissemination, using VANET.

RETRACTED

The purpose of the this study is to develop an enhanced VSL strategy called Intelligent Advisory Speed Limit Dedication (IASLD) that exclusively determines the advisory speed limit of each vehicle based on the vehicle safety capability in addition to the traffic and weather condition. The utilization of this approach leads to improvement in traffic flow, reduction in travel time of vehicles, and acceleration in procedure of congestion detection, in comparison with the current traditional VSL approaches which are using loop detectors. The IASLD as an integrated VSL system employs the mounted cameras, sets of loop detectors, and RSUs for its operation along the highway.

The rest of the paper is structured as follows. In Section 2, an overview of existing VSL systems and factors that affect VSL systems is described. In Section 3, we introduce IASLD architecture. In Section 4, we described our study network and results and evaluations are also explained in the same section. Finally, Section 5 concludes the paper and highlights the findings. To understand the definitions of acronyms please refer to Table 1.

## 2. Variable Speed Limit System Overview

### 2.1. System Description

The general framework of the VSLs includes employment of several sensors installed along the highway which divide the highway into different monitoring segments. The procedure of decision making about the advisory speed limits is done by taking advantage of the information obtained from these sensors, exclusively for each segment of the highway. Furthermore the VSL includes variable speed limit signs, VMS, and a central processing unit to perform control actions.  Figure 1 shows utilization of VLS to update drivers of the road condition ahead and to display the current speed limit based on the VSL control strategies.  Figure 1 depicts a three-lane highway equipped with loop detector stations, spaced 500 m apart. The detectors obtain traffic information including speed, occupancy, and count; then the VSLs display a proper speed limit for drivers, based on the traffic information received from loop detector.

### 2.2. VSL Strategy

Effectiveness of VSLs is vastly dependent on the VSL control strategy utilized (e.g., circumstances under which speed limits are increased and decreased), level and type of enforcement, and the traffic conditions [10] in the manner that proper control strategy in installation of the VSL systems can lead to enhancement in driving safety of 30 percent [11].

RETRACTED

Existing VSL switching follows simple rule-based control strategies, in which real-time decisions are made based on predefined thresholds of traffic flow, mean speed, or occupancy (i.e., the percentage of time during which the loop detector occupied) received in a periodic manner from the loop detector. The main framework of current VSLs is specifically involved with detection of occupancy exceeding the specific threshold (~15%) or volume exceeding the predefined threshold (~1600 vphpl) according to the vehicles' speeds in highway. Amongst, the VSL system implemented in the M25 controlled highway in the UK [12] activates once the loop detector perceives the segment's volumes exceeding 1650 vehicles per hour per lane; therefore, the segment's speed limit reduces to 95 km/h from the default of 112 km/h. The A2 controlled highway in Netherlands [13] is another example of VSL implementation in which VSLs reduce to 90 or 70 km/h by considering volume and speed data achieved by loop detector station in every 1 minute interval. Abdel-Aty et al. [11] developed VSL control algorithm which chooses a suitable speed limit based on measurement of average station volume, occupancy, and average speed of vehicles received in a periodic manner (20 s) from the loop detector. Authors performed several modifications to thresholds of VSL detection parameters, to evaluate improvement of safety as the matter of CP, overall highway congestions, and reducing the growth of travel time.

The structure of VSL control strategy for providing the proper speed limit of vehicles according to proposed VSL approaches is depicted in Figure 2. This structure solely considers the occupancy, volume, and average speed of vehicles as VSL decision making criteria.

Despite consideration of three traffic parameters in this structure, the average speed is the parameter which itself is affected by the volume and does not have significant role as criterion of instant traffic controlling. In addition, there are other significant criteria that need to be considered. Meanwhile the adverse weather condition is one of important factors affecting traffic road safety and fluency. Driving during adverse weather is counted to be hazardous in the condition of ignoring the safe speed limit. Recent study by Andrey [14] showed that 5% of road casualties in Canada are tied directly to the weather. It was also found that winter storms bring a superior hazard of being involved in a crash by as much as 25 times—greatly superior than the increased hazard brought by behaviors that state governments already have placed sanctions against, such as speeding [15]. Thereby many authors [15–18] assess the speed management in inclement weather in order to improve traffic safety in such conditions. Ewan et al. [18] investigated the reliability of utilizing weather sensors for variable speed limit system. Authors experimented reliability of data under various surface states in a controlled laboratory environment. However, the results showed accuracy in some surfaces, and readings of some others were highly inaccurate. Martí et al. [16] proposed a method to check the value of data achieved by weather sensor in order to improve the quality of the taken decisions by the system.

RETRACTED

Beside road and weather conditions, vehicle safety capabilities have a dramatic impact on vehicle stability and controllability which have not been studied despite decades of working on VSL control strategies. All in all, to the best of our knowledge, there have been no approaches proposed that address all the aforementioned criteria comprehensively in VSL decision making strategy.

### 2.3. Factors That Affect the VSL Impact

The effectiveness of VSL systems is highly sensitive to driver compliance. Therefore, evaluation of VSL is affected by the level of driver compliance which might vary under different traffic circumstances. Hellinga and Mandelzys [10] and Lee and Abdel-Aty [19] utilized microscopic simulations to evaluate the sensitivity of the operational impacts of VSL to driver compliance. Cameron and Duncan modeled several scenarios for four degrees of compliance (i.e., low, temperate, high, and extremely high) using the PARAMICS microscopic traffic simulator [20]. Findings of the simulator experiment indicated that safety benefits of VSL in extremely high compliance scenarios are four times more than the benefits achieved in the low compliance scenarios. Lee et al. studied the effects of different warning messages and VSLs on driver compliance by observing behavior of 86 participants. The study showed that compliance rate varies under different types of message posted on DMSs. Further analysis by Zhao et al. [21] indicated the degree of trust in DMS (e.g., road information and speed limit) and the familiarity with road network has significant effect on the level of driver compliance.

Since the overstep from speed limits by drivers can depend on trust of them to the vehicle characteristics, it seems to be needed to consider more realistic VSL system that allocates the reliable advisory speed limits on the basis of engineering principles which are involved with vehicles featuring. Many drivers, who ignore the regulatory or advisory speed limit in highways, believe that posted speed is low for their vehicle [22]. We believe the degree of trust can be improved if drivers ensure that the speed limit control system considers the vehicle characteristics such as vehicle type, weight, size, and safety capabilities, in addition to all other conditions (i.e., road and weather). To the best of our knowledge, despite decades of working on VSL systems, no such system has been found to date. Therefore, applying the IASLD as a VSL system which considers the important factors related to driver's point of view can increase the level of driver compliance.

RETRACTED

## 3. Intelligent Advisory Speed Limit Dedication (IASLD)

IASLD is an enhancement of VSL systems which primarily aims to optimize the traffic flow, traffic safety, and travel time of vehicles, in highway scenarios in an innovative manner. The prominent preference of IASLD with proposed VSL systems is the essence of comprehensive multiprocessing of the circumstances which have direct effect on VSL decisions. The IASLD takes advantage of integrated framework to prepare the advisory speed limit for each vehicle exclusively in successive segments of the highway. The road condition, traffic flows, incident occurrences, vehicle's type, and vehicle's safety capabilities are the factors which have significant role in decision making of the IASLD. Another prominent feature of IASLD is taking advantage of VANET technology for its information propagation.  Figure 3 illustrates general overview of IASLD performance. As it is depicted, there are sets of RSUs and loop detectors which are deployed at identical distances of the highway. Deployment of these two instruments makes the highway monitoring into several segments which require consideration of different advisory speed limits according to the governed circumstances in that particular area. In addition there are sets of mounted cameras in the middle of each monitoring area. These cameras have the responsibility of detecting the plate number of vehicles which are crossing them. The IASLD by utilizing the proposed approach in this study calculates the exclusive advisory speed limit for each vehicle crossing the camera for the following area and sends it to the vehicle when it reaches to vicinity of the RSU which is at the beginning point of the following area. The succeeding subsections deeply clarify the procedures of highway condition detection, vehicle identification, advisory speed limit calculation, and advisory speed limit propagation in IASLD.

### 3.1. Highway Condition Detection

#### 3.1.1. Road Condition

Weather conditions have a considerable impact on the safety and operations of the highway transportation system. Road weather sensors are frequently utilized as part of RWIS stations as a feasible tool for monitoring the road conditions in severe weather conditions [18, 23]. These sensors fall into two main types, namely, in-pavement and noninvasive. Improvements in road weather sensing technologies have made noninvasive road weather sensors a precious module in various ITS applications. Ewan et al. [18] investigated the reliability of these sensors for weather-responsive VSL systems. Authors found the Vaisala remote surface state and temperature sensors (DSC-111 and DST-111) and determined the surface states such as dry, wet, snowy, and icy accurately and reliably. Note that in this study we assume weather data is already collected by such sensors; therefore, here we are not going through focusing on how weather data is obtained. In this study, we focus on the road conditions that can be obtained from the sensors including dry, wet, and icy.

RETRACTED

#### 3.1.2. Traffic Flow Condition

The increasing demand of the driving public for exact traffic data has spurred the deployment of dedicated monitoring systems that primarily consist in employment of point sensors. This type of sensors such as inductive loop detectors and video cameras provides inexpensive solutions for obtaining fairly accurate traffic information [24].

Inductive loop detectors are enormously installed on highways worldwide, with enlarged utilization since early 1990s, where densities reach one detector in almost every 500 m [25]. Loop detector stations are embedded in the pavements along a highway in order to monitor congestion and to provide information for traffic control operations. These detectors are presence-type detectors which are able to detect the presence of a metallic object above them. Nowadays, dual loop detectors, which consist of two closely spaced wired, are commonly used. Loop detectors collect speed, volume, and occupancy data at a specific time interval (regularly 15 to 30 seconds) for each lane at the detector site by the road side detector controller in order to compute the flow average. Accordingly the parametric values for the control algorithm of current work are chosen on the basis of aforementioned engineering principles. In IASLD we consider two different congestion categories named light congestion and moderate congestion. The volume of 1800 vphpl or occupancy threshold of 14.8% is specified for detection of light congestion and volume threshold of 2000 vphpl is specified for detection of moderate congested as mentioned in the Highway Capacity Manual 2010 [26, 27] for three lanes highway.

RETRACTED

#### 3.1.3. Incident Detection

In recent decade, there have been various studies on detection of different types of incidents in highways using the VANET technology [28–31]. Such approaches have constantly followed two different aims from the matter of traffic controlling: (1) using CCWS to detect the incident by the probe vehicle which encountered the incident and warn it to the rear drivers who are in the specific hazard zone close to the incidents to prevent from chain collisions [32, 33]; (2) using the IDS to perceive the occurrence of incident in the specific zone and applying the necessary traffic controlling actions along the highways. The utilization of IDS commonly has been involved with employment of infrastructures beside the highway to obtain and process the data sent from the probe vehicles as the incident detectors and afterwards proceed the safety actions for controlling the traffic and hence the incident detection procedure of IASLD places in this category.

For the IDS there have been different approaches proposed to make efficient incident detection through the highways. In [34, 35] authors proposed the consideration of speed acceleration of vehicles by using kinematics data and mobile sensors, respectively. Thus, the deceleration of vehicles in specific point and then their acceleration to normal velocity after passing that specific point are assumed as occurrence of incident. In [36, 37] authors proposed consideration of the travel time of vehicles while crossing the specified zones to determine the traffic condition and detect the incident. In [37] authors suggest the comprehensive CCWS which consider the combination of aforementioned detection criteria including the inspection of vehicles travelling time on the supervised highway segments and considering the speed acceleration in addition to lane changing behavior of cluster of vehicles at specific zones. In [38, 39] authors suggest using EDR as vehicles' on-board devices which have the responsibility of recording the lane changes along the specified highway segments and sending the information when vehicles reach to vicinity of RSU. RSU will have the duty of processing the obtained data including the density of vehicles in specified segments and their lane changing behaviors considering the algorithm named Bayesian to compute the posterior probability of incident occurrence. In addition, authors have considered the driver intervention as an option of informing the traffic controller about existence of any incident.

In IASLD, we were looking for an approach to be more fitted into its characteristics as a matter of fading out the aforementioned literatures' limitations: (1) requirements for placing the vehicle in vicinity of RSU and passing nearby the RSU to transfer the motional data which will not be competent in the congested conditions; (2) deficiency of considering the lane changing in the circumstances in which all the road width becomes obstructed; (3) lengthy time period for aggregation of motional data and assessing them in RSU, which causes loss of the great deal of effective time for safety signaling and controlling the traffic; (4) in addition, in all of the aforementioned literatures, there is necessity of evaluating the movement condition for cluster of vehicles to make reliable decision about incident detection.

RETRACTED

In our approach similar to majority of previous related works, we assume all the vehicles travelling in the highway are equipped with OBU for computing the motion state of vehicle in addition to decision making on the signal transmission between vehicle and infrastructure. Furthermore we assume all the vehicles use wireless transceiver and GPS including the digital map. All the communications defined in WAVE spectrum and communication between vehicles and infrastructure RSUs are available all over the highway road.

We assume the detection of incident at any location of the highway as the sudden deceleration of vehicles due to the instant reaction of driver for avoiding the hazard. This deceleration may be regarding the existence of breakdown or accident or any other types of incident. Our consideration for measuring the vehicles emergency stopping deceleration according to the three seconds safety stopping distance in ITS literatures [40] is 9 m/s^2^. This amount is the deceleration considered for vehicle when it makes sudden break and reduces its velocity dramatically and hence OBU by detecting the equal and further values of 9 m/s^2^ deceleration broadcasts message (packet) called incident warning message to inform the RSU about its sudden deceleration. The structure of incident warning message is shown in Figure 4.

In this structure, the “vehicle ID” is the ID of the vehicle as the origin of sending the packet which is defined as the plate number of the vehicle. The “unique event ID” specifies the type of the message; this filed is used to discern the incident warning message from other types of messages which are sent through the highway. The “position coordination” specifies the 2D coordination (latitude longitude) for specifying the location of event for subsequent operations of traffic controller and finally the “message sequence number” is defined for assisting the RSU infrastructure in identifying the different incident warning messages which may be sent by the same vehicle.

RETRACTED

The vehicle which has detected the 9 m/s^2^ deceleration broadcasts the incident warning message periodically according to the specified beacon generation rate up to the time it receives the acknowledgement packet from the RSU as a confirmation of receiving its data. The deployment of the RSU infrastructures along the highway is in the way that it makes the full coverage of the WAVE propagation for detecting the messages by either RUSs or vehicles. This layout is illustrated in Figure 5.

### 3.2. Vehicle Identification

#### 3.2.1. Classification

Employment of USL for existing VSL systems, in which speed limits are same for all types of vehicles, is inappropriate to account for all potential safety issues. The size and weight differences between passenger cars and heavy vehicles and special maneuverability characteristics associated with these two types of vehicle imply on considering more distinctive speed limits for different types of vehicles. Hence, it is required to take advantage of DSL strategies to address this issue [41].

DSLs for trucks and cars are becoming a promising way to enhance highway operation and safety. Thus, in this study we focus on DSL strategy which restricts vehicles with specific size and weight, to travel at lower speeds than the rest of the traffic stream [42], as heavier vehicles require a larger stopping distance and stopping time than do passenger cars [43]. Thereby, vehicles are divided into three types based upon their capacities. Note that capacity measurement for heavy vehicles such as trucks is not determined based on the number of passengers; therefore, capacity does not necessarily mean the number of vehicles' passengers. The capacity of maximum number of 8 passengers (up to 1500 kg) for first type, maximum number of 15 passengers (up to 2500 kg), and over 26 passengers (over 2500 kg) for second and third types, respectively, is considered for vehicle classification. Each type is divided into two classes termed class “A” and class “B” vehicles that include vehicles with modern braking systems and vehicles with traditional braking systems, respectively. Braking regulations are varied among different countries; for instance, ABS compliance with directive 17/320/EEC is mandated in Ireland since April 2009 for all types of vehicles and correspondingly in UK since July 2004 [44]. Hence, vehicles produced before April 2009 in Ireland are counted as class “B” and newer is considered as class “A” vehicle. Since main objective of this study is movement safety of vehicles along the highway, the IASLD concentrates on vehicles' type in addition to the producing year of vehicles (considering the braking regulation) as a key parameter for measuring safety capabilities.

RETRACTED

#### 3.2.2. Safety Capability

In IASLD, consideration of vehicles' classification, beside their safety capability, leads us to defining different safe speeds for the current road condition. The vehicle's safe speed determination starts by employing default speed limit specified for different locations of highway, and then safe speed will be defined more specifically by considering vehicle weight, size (utilizing the vehicle classifications), and safety capabilities (e.g., braking systems including the ABS, EBD, ESP, etc.) that are varied among different vehicles. This means that the safe speed for vehicle with the higher safety capability is higher than vehicle with lower safety capability. For instance, safe speed is higher for vehicles equipped with ESP, EBD, and/or ABS. The reason is that such equipment increases the vehicle stability, controllability, and braking efficiency, as a result, leading to reduce the stopping distance as shown in Figure 6. More detailed information on differences between braking with EBD/ABS turned ON and OFF is available in [45, 46].

The SSD for various vehicles can be obtained from (1); in this equation the *D*_*p*−*r*_ measures the perception-reaction distance [47] and the *D*_braking_ measure the braking distance:

(1) $$\begin{array}{c} D_{p-r}=1.4\nu \cdot t,\;\;D_{\text{braking}}=\frac{\nu^{2}}{2g\left(\mu \pm G\right)},\\ \text{SSD}=D_{p-r}+D_{\text{braking}}=1.4\nu \cdot t+\frac{\nu^{2}}{2g\left(\mu \pm G\right)}. \end{array}$$

In *D*_*p*−*r*_ the *ν* represents the velocity of vehicle and the 1.4 is the constant coefficient to account for dissimilarity in the height of the driver's sight and height of the obstacle. Moreover, *t* shows the reaction time interval of the driver until starting the braking. As an average, *t* is considered as 1 second for mature drivers. However, as a general reliable time of reaction considering the elderly and immature drivers this value is considered as 1.5 seconds. In *D*_braking_ the *g* value specifies the gravity of earth and *G* defines the gradient coefficient of the road which can differ depending on either road uphill or downhill structure. In our study, we assume the value of *G* as 0. The parameter *μ* in *D*_braking_ represents the friction coefficient which can differ by classification of vehicles (three different classifications) in addition to their safety capability for each road condition (dry, wet, or icy). This variable can be obtained from (2) in which the TW variable specifies the tread wear of the vehicle and it can differ by equipping the vehicle with ABS and EBD systems as a single variable which affect the calculation of *μ*

(2) $$\begin{array}{c} \mu =\frac{2.25}{{\text{TW}}^{0.15}}. \end{array}$$

Since in this study our concentration is not on the details of friction coefficient calculation, we assume different values of *μ* for obtaining the safe speed of vehicles in each road condition. Note that these values have approximate entity and can be slightly modified depending on the local conditions of tires and roads which are employed in any specific area. Hence, we have considered the average value of friction coefficient for the vehicles, by taking advantage of the information provided in [48–50].

RETRACTED

In this approach for obtaining the safe speed limit of vehicles we merely focus on the *D*_braking_ as the main parameter that influences the SSD of vehicles. We dispense the parameter *D*_*p*−*r*_ owing to similarity of driver reaction times in same speeds. We specify two baselines as standards respectively for vehicles with less than 2.5 ton weigh (types 1 and 2) and for vehicles with more than 2.5 ton weigh (type 3), to suggest the different safe speed limits in highways. In this matter we take advantage of safe vehicle headway standard of three seconds introduced in [40] to make sure about the efficiency of our baselines. The first SSD baseline defined as the distance takes for the passenger vehicle with the friction coefficient of 0.9 in its current default speed of the highway (100, 80, 60, or 40 km/h). Using the mentioned values for *D*_braking_ provides the first SSD baselines depicted in Table 2. The second SSD baseline defined as the distance takes for the heavy vehicle with the friction coefficient of 0.45 in its current default speed of the highway (70, 60, or 40 km/h). Using the mentioned values for *D*_braking_ provides the second SSD baselines depicted in Table 2. We discuss further in the “advisory speed limit calculation” subsection the consideration of various default speeds in different parts of the highway.

Using the SSD baseline values (which vary depending on the current default speed of the area in highway) in addition to friction coefficient of different types of vehicles in various road conditions aids us to calculate the safe speed for different types of vehicles using (3). Hence, Table 3 indicates the various values of friction coefficient for obtaining the safe speed according to the classification and safety capabilities of vehicles in three different road conditions. In this measurement we have considered the safety capabilities of vehicles into two classifications; the first classification comprises the vehicles which are equipped with modern braking systems (ABS/EBD/ESP) and the second classification comprises the vehicles which are not getting assistance from the modern braking systems and safety capabilities

(3) $$\begin{array}{c} \nu =\sqrt{\text{SSD}\times 2g\left(\frac{2.25}{{\text{TW}}^{0.15}}\pm G\right)}=\sqrt{\text{SSD}\times \left(2g\mu \pm G\right)}. \end{array}$$

Availability of aerology data as the road condition and the information of vehicle classification enables the IASLD to offer the safe speed limit for each vehicle according to the current default speed limit of the highway using Tables 2 and 3 and (3).

RETRACTED

#### 3.2.3. Vehicle Recognition

Vehicles' type should be identified for proper classification based upon their characteristics. To accomplish this goal, vehicle model is recognized by detecting the vehicle's license plate using series image processing techniques. To do so, frontal view vehicle image is first transformed to grayscale with 8-bit resolution and then scaled to 640 by 480 pixel size, and after that a LPR module is performed. An adaptive image segmentation technique SCW [51], which uses image statistics such as standard deviation and mean value as a heuristic for possible plate location, utilizes for LPR. LPR also uses masking and binarization with sauvola method [52], followed by connected component labeling and binary measurements.  Figure 7 depicts some steps of the LPR while Table 4 highlights the pseudocode of the license characters recognition which initiates by cropping the specified coordination (defined in matrix A) of last plate segmentation step. The entire process is reasonably fast on average which is about 100 ms.

The LP candidates considered in plate location stage are examined in the phase of character segmentation which takes place once plate localization is developed. In order to isolate characters in the license plate image, license plate preprocessing is performed. Considering a candidate region, the specific coordinates are evoked for cropping the particular subimage. By utilizing the bicubic interpolation method, this image is converted to a standard size (77 × 228 pixels) and then exposed to the SCW segmentation method with the following parameters: *X*_1_ = 2,  *Y*_1_ = 5,  *X*_2_ = 4,  *Y*_2_ = 10, and *T* = 0.7, where the measurement is the STD value. Selecting the mentioned parameters is explained by [51]. Following the inversion and resulting image and object labeling, the orientations and heights of connected components are then calculated. The objects whose measurements do not fulfill specified rules (orientation > 75° and height > 32 pixels) are removed.

The remaining objects are then forwarded to a trained PNN where maximum matching probability with the database class for the best match is provided. The main advantage of utilizing a PNN is training and classification speed that is proper for real-time applications. The PNN is based on the Bayesian classifier:

(4) $$\begin{array}{c} P\left(\frac{c_{i}}{x}\right)=\left(\;\frac{P\left(x/c_{i}\right)P\left(c_{i}\right)}{\sum_{i=1}^{n}p\left(x/c_{i}\right)P\left(c_{i}\right)}\right), \end{array}$$

where *P*(*x*/*c*_*i*_) is the conditional probability density function of *x* given set *c*_i_, *P*(*c*_*i*_) is the probability of drawing data from another class *c*_*i*_, Vector *x* belongs to class *c*_*i*_, and if *P*(*x*/*c*_*i*_)  >  *P*(*x*/*c*_*i*_), *j* = 1, 2,…, *n*,  *j* ≠ *i*. PNN approximates the probability that vector *x* belongs to a particular class *c*_*i*_ (i.e., it estimates the likelihood of an input feature pattern being part of learned category) as a sum of weighted Gaussian distribution centered at each training sample given by

(5) $$\begin{array}{c} \frac{1}{\left(2\pi \right)\left(p/2\right)\sigma^{p}N_{i}}\;\overset{N_{i}}{\underset{j=1}{\sum }}\exp\frac{-\left(x-x_{j}^{i}\right){\left(x-x_{j}^{i}\right)}^{T}}{2\sigma^{2}}, \end{array}$$

where *x*_*j*_^*i*^ is the *j*th training vector for patterns in class *i*, *σ* is the smoothing operator, *N* is the dimension of the input vector, and *N*_*i*_ is the number of training patters in class *i*. For nonlinear decision boundaries, the smoothing operator *σ* requires being as small as possible. Otherwise, the designed network takes into account several nearby design vectors. Authors in [51] reported achievement of 96.5% success rate in plate segmentation and 89.1% for the recognition of the entire plate content in above modules.

RETRACTED

One of the novelties of the present study is to employ a hierarchical database to reduce the recognition time. This database includes a set of smaller databases, per vehicles' manufacturers, with all the vehicles' types and safety capabilities (class A and class B) as depicted in Figure 8.

### 3.3. Advisory Speed Limit Calculation

According to what mentioned hitherto in IASLD, we need to propose an integrated framework for suggesting the advisory speed limits. This framework must manipulate all the mentioned environmental occurrences which have effect on IASLD decision making. Hence, initially, we go through defining the default speed limits of highways which have to be considered according to the traffic conditions of the highway and afterwards we discuss the IASLD framework for suggesting the vehicles' advisory speed limits.

In IASLD the highway is divided into equal-length segments. For each segment, there are two default speeds defined for vehicles; the first default speed is concerned with the first and second types of vehicles and the second default speed is concerned with third type of vehicles as heavy vehicles. The procedure of decision making on the default speeds of each segment is dependent on the current traffic condition in the highway. Hence at the outset we go through the computation of default speeds for each segment.

RETRACTED

In IASLD the default speeds of the vehicles in an ordinary condition which is not involved with any traffic restriction are considered as 100 km/h (~60 mph) for the first two types and 70 km/h (~40 mph) for the third type; these values are the standard speed limits proposed for most of urban highways [53, 54]. In IASLD the segments with ordinary speed limit are called regular area.

Using the IASLD system along the highways aids us to detect three types of traffic congestions along the highway. These detections comprise the heavy congested, moderate congested, and light congested traffic flows, which is concerned, respectively, with detection of incident in specific segment of highway, the detection of either volume threshold of 1800 vphpl or occupancy threshold of 14.8% by the loop detector in specific location of highway, and finally the detection of volume threshold of 2000 vphpl using the loop detector.  Figure 9 illustrates the three types of traffic congestions and their restricted speed buffering along the highway. As it is depicted, the heavy congested traffic flow is defined by detection of incidents in specific segment of highway by taking advantage of VANET. The detection of heavy congested condition in specific segment leads the IASLD to define four subsequent segments of highway including the congested segment and its three prior segments as the restricted area. In IASLD the restricted area is the area with limited default speed for vehicles, in comparison with regular area. From the other side, the detection of moderate and light congested condition using the loop detectors leads the IASLD to define, respectively, three and two successive segments of the highway—including the segment ahead of the loop detector and its prior segments, as the restricted area. As it is depicted in Figure 9, in each traffic condition the default speed limit of restricted areas varies by the distance of their segment from the congested area. In addition, it is worth mentioning that in IASLD the restricted areas can be extended in case any traffic congestion detected again along the restricted areas; thus, the restricted areas will be redefined and reiterated again from the point of detection.

By defining the default speed limits of regular areas and restricted areas for different segments of the highway, the framework of IASLD advisory speed limit calculation can be illustrated as Figure 10. This framework operates as follows.

RETRACTED

For each vehicle driven in the highway prior to reach the subsequent segment, the IASLD calculates its advisory speed limit for the upcoming segment. Hence, in the first phase, the IASLD checks whether there is any collision detected along the highway. If so, it checks whether the following segment is among the restricted areas of heavy congestion. In case it is verified, the default speed restriction (according to the restricted area that vehicle is going to be placed on) will be stored as the 1st restriction in the system. In the second phase, the IASLD checks in case there is any traffic congestion including the light or moderate congestion detected in the highway, whether the following segment is among the restricted areas. If it is verified that the default speed restriction will be stored as the 2nd restriction in the system. In the third phase, the IASLD goes through the vehicle identification phase by doing the license plate recognition and PNN matching for identifying the vehicle classification from the database. Two processes of vehicle classification recognition and safety capability identifications will be done by utilizing the plate number capturing and database adaption during this phase. In the fourth phase, the IASLD goes through the election of appropriate friction coefficient according to the vehicle classification, vehicle's safety capability, and current road condition using Table 3. In the fifth phase, IASLD checks whether there is any speed restriction stored in its buffer, including the 1st restriction and 2nd restriction. If yes, the minimum speed restriction will be chosen as the default speed restriction for the upcoming segment. In case there is no speed restriction, the IASLD will consider the regular area default speed for the upcoming segment. In the final phase, the IASLD calculates the advisory speed limit for the vehicle according to the friction coefficient obtained from the phase four and the SSD baseline obtained according to the chosen default speed from the Table 2.

### 3.4. Advisory Speed Limit Propagation

The abilities of VANET have caused it to become a suitable network consisting the multipurpose characteristics for superfluity of applications [55]. The proposed VANET-based applications in ITS can generally classify into two main categories on the basis of their provisioning services, either providing the infotainment services or providing the safety related services [56]. The infotainment services comprise traffic information, advertisements, video streaming services, and so forth; from the other part, the safety related services comprise lane closure information, CCWS, and generally other types of urgent incident informing systems. The infotainment services have less stringent on delay requirements in comparison with safety related services. Thus in IASLD the advisory speed limit propagation is placed in the first category, which can tolerate seconds of delay.

RETRACTED

The procedure of information dissemination for infotainment services has predominantly been involved with usage of broadcasting [21]. The reason for choosing this method of propagation is the public-interested essence of such information for specific ROI. Hence there have been varieties of approaches proposed with aim of increasing the performance of information broadcasting from RSU to vehicles in their proximity for highways. Such works regardless of their dissemination procedure have concentrated on increase of transmission rate and supported distance by either usage of multihop broadcasting [57, 58] or usage of single-hop transmission of broadcast messages [59, 60]. The characteristics of IASLD as a system with capability of propagating the different exclusive advisory speed limits for vehicles lead us to modify the procedure of information propagation to unicast dissemination of messages for each vehicle. The procedure of IASLD advisory speed limit propagation is as follows.

This procedure starts by broadcasting the beacon messages from each RSU; thus each RSU infrastructure broadcasts this packet periodically (using fixed beacon generation rate) to inform the vehicles in vicinity of RSU about its existence. The considered procedure of beacon message propagation in IASLD is one-hop broadcasting. The reason of choosing this type of broadcasting in IASLD is creating the direct communication between the vehicles placed in short distance (proximity of maximum 150 m) to the RSU and making low latency due to the absence of intermediaries [61]. The structure of RSU beacon message is depicted in Figure 11.

In this structure the “RSU ID” specifies the ID of RSU for further communication of vehicles and the “unique event identifier” specifies the type of the message for differentiating the RSU beacon message used for advisory speed limit propagation with other type of beacons that vehicle may receive. The “area coordination” specifies the 2D coordination (latitude longitude) of start point and end point of the area (segment) that RSU is going to offer its advisory speed limit. The vehicle's OBU which receives the beacon message with specified unique identifier firstly checks whether it exists in the distance of 150 m from the termination of its current advisory speed limit area; if yes, it replies request message to the RSU using the RSU ID. The structure of advisory speed limit request message is shown in Figure 12.

RETRACTED

In this structure the “vehicle ID,” “unique event ID,” and “RSU ID” have the same aforementioned attributes. The “plate number” field specifies the plate number of vehicle. This field assists RSU to learn the vehicle ID according to vehicle's plate number for further sending of advisory speed limit to that specific vehicle. By receiving the request message from vehicle, the RSU matches the vehicle's plate number with calculated advisory speed limit obtained from previous section (Figure 10) and sends the advisory to the vehicle. The advisory speed limit message structure which sent as one-hop unicast propagation is illustrated in Figure 13.

In this structure, the “advisory speed limit” filed presents the exclusive advisory speed limit calculated for the vehicle, and “area coordination” field specifies the start and termination point of the area in which the advisory speed limit is defined and vehicle is going to enter in. The RSU sends the advisory speed limit message periodically (using fixed generation rate) up to the time it receives the acknowledgement packet from the vehicle as a confirmation of receiving the advisory speed limit message.

The reason of using one-hop propagation of packets in our scenario is suitability of one-hop propagation for delivering the information to the vehicles which are in close vicinity of the RSU and in the view of the fact that advisory speed limit propagation is used merely for vehicles which are crossing from one monitoring segment to another.

## 4. Study Network Description and Assessment

The considered environment for applying the IASLD architecture is 8 km section of the Klang highway located close to Kuala Lumpur, Malaysia. The Klang highway has three mainline lanes, containing three interchanges as shown in Figure 14. The concentration of evaluation is on the movement direction from coordination of 3.103235, 101.585318 heading to northeast of highway. The default speed limit specified for vehicles is 100 km/h for passenger vehicles and 70 km/h for heavy vehicles. The selected route includes three interchanges and consists of negligible dual-loop detectors in specific zones which have high potential of unexpected congestions. In this approach, we have taken advantage of SUMO traffic simulator [62] for simulating aforementioned area of the highway. The highway area is split into 500 m monitoring segments by dual-loop detectors that are placed beside APs. In addition, highway cameras are mounted in distance of 250 meters to the loop detectors. Information about traffic conditions and vehicle image captured by cameras is sent to traffic controller. The considered distance between mounted cameras and RSUs verifies the time interval required for the traffic controller for detection and preparation of advisory speed limit by the time vehicle reaches the vicinity of RSU.

RETRACTED

### 4.1. Simulation Study

For testing and evaluating the IASLD simulations, we have used the NS-2.34 [63] and SUMO by taking advantage of TraCI [64] for interconnecting them. The interconnected simulation of traffic and network scenarios produces realistic simulations of VANET which is adapted to our approach. TraCI utilizes TCP-based client/server architecture which makes SUMO and NS-2 to update information in real time. The focus of simulation setup and evaluations in this section does not cover the vehicle recognition procedure as plate number detection owing to usage of virtual simulation environment. Hence, we assume that the information of vehicles according to their plate number is already prepared for traffic controller.

#### 4.1.1. Traffic Simulation Setup

SUMO traffic simulator is highly portable microscopic traffic simulator which is chosen to create the Klang highway traffic scenario. Thus, we considered aforementioned characteristics of Figure 14 including three entrances and exit points along the highway. Table 5 indicates the parameters utilized for modeling traffic environment beside network operation. Three types of vehicles are deployed 75%, 20%, and 5%, respectively, for passenger, van, and heavy vehicles. The portions of safety capabilities for each vehicle's type are 70 and 30 percent for classification A and B, respectively. Accordingly, the friction coefficient values of Table 3 are configured for simulating different degrees of stopping distances in dry, wet, and icy road conditions. Drivers may accelerate or decelerate according to the specified speed limits of the highway. The chosen speed of the vehicles by drivers is between 80% and 110% of the legal speed limits which is defined by taking advantage of attribute speedFactor and speedDev to achieve realistic traffic behavior. The impatience value which represents interest of driver for using the gaps in the sense of collision avoidance for changing lane is considered as 0.8. This value implies the average level of driver compliance which we have considered for making the highway traffic scenario more realistic. The deceleration of 9 m/s^2^ is configured as emergency deceleration which defines occurrence of incidents. The maximum number of 400 vehicles is utilized for obtaining the volume of 1600 vphpl in the highway simulation. In addition, the concentration of evaluation is confined to the middle 6 km of the highway to eliminate border effects.

RETRACTED

#### 4.1.2. Network Simulation Setup

The configuration of NS-2.34 network simulator is as follow: all the parameters for PHY and MAC layer communications are defined in IEEE 802.11p spectrum [65] using 6 Mbps data rate and QPSK modulation with 5.9 GHz frequency. The maximum supported communication range is defined as 300 meters, using the transmission power of 16.8 dB_m_ and 10.8 dB_m_ for RSU and vehicle, respectively. TwoRayGround radio propagation model is utilized to obtain realistic simulation of radio propagation in highway scenario. This propagation model considers direct line of sight between transmitter and receiver in addition to ground reflected propagation path which constitutes the most signal attenuation of highways. The consideration of environmental noise is only limited to the thermal noise with value of −104 dB_m_ due to negligibility of external sources of noises in 5.9 GHz frequency. The chosen length of packets for incident warning message, RSU beacon message, advisory speed limit request message, and advisory speed limit message are 250, 100, 200, and 250 bytes, respectively. The packet generation rate is chosen as 5 Hz, at which 5 beacon messages broadcasted every second. The overview of parameters utilized in Network simulator is depicted in Table 5.

#### 4.1.3. Results and Evaluations

Evaluation of this study encompasses the comparison of IASLD performance with VSL and Non-VSL approaches. The performance assessments mainly include consideration of travel time, traffic flow, and occupancy in different traffic scenarios (light, moderate, and heavy congestion). Moreover, the impacts of IASLD, VSL, and Non-VSL approaches are tested under different road conditions (dry, wet, and icy). The VSL control strategy utilized in the present evaluation is referred to in Figure 2. Moreover, Non-VSL approach contains static consideration of 100 Km/h and 70 Km/h for passenger vehicles and heavy vehicles, respectively, along the highway.

Figure 15 illustrates the impacts of IASLD, VSL, and Non-VSL strategies on travel time under three different road conditions. In particular, this figure depicts the average travel time taken for vehicles in each of the approaches at the successive 500 meters distances of the selected highway. The results are split into three clusters of dry, wet, and icy road conditions. Simulated traffic condition has been free of congestion with the average volume of 1430 vphpl, 1120 vphpl, and 311 vphpl in dry, wet, and icy conditions, respectively. The results indicated evident superiority of IASLD in comparison with VSL from the matter of reduction in average travel time for the distance above 2500 meters, in a way that IASLD has achieved 9.3%, 6.4%, and 2.9% improvement, respectively, in dry, wet, and icy conditions. Moreover, the essence of multifarious consideration of speed limits in IASLD in dry condition has led to improvement of travel time in comparison with Non-VSL approach in some cases, so that the average travel time of IASLD is 4.4% less than Non-VSL after 8000 meters travelling. This preference was not observed in icy and wet conditions owing to absence of real-time restriction in displayed speed limit.

RETRACTED

Figure 16 clarifies the impacts of IASLD, VSL, and Non-VSL strategies on average volume under three different road conditions. The graphs represent the average volume of traffic detected in entire time of simulation run in consecutive locations of the highway. This experience was done by using 230, 160, and 70 vehicles for dry, wet, and icy conditions, respectively. The presence of exits prior to stations 20, 80, and 160 caused notable decline in average volume of the vehicles detected from these stations. In addition, the presents of entrances before stations 30 and 90 led to dramatic increase of detected average volume. The results showed that the average volume of the vehicles under dry condition has been 1304.89, 1320.92, and 1356.01 for Non-VSL, VSL, and IASLD approaches, respectively. Furthermore, the average volume under wet condition has been 953.174, 961.71, and 985.7 for Non-VSL, VSL, and IASLD approaches, respectively. Moreover, the average volume under icy condition has been 262.22, 271.4, and 285.14 for Non-VSL, VSL, and IASLD approaches, respectively. Providing the higher range of reliable advisory speed limits for eligible vehicles in IASLD has caused apparent increase in volume of vehicles that are travelling along the highway which means, by considering the equality of number of vehicles in all the three approaches, the IASLD utilization had led to more fluency of vehicles movement. The ratio of differences between average volume of IASLD, VSL, and Non-VSL has had gradual reduction under dry, wet, and icy conditions, respectively. This is owing to the fact that results showed that the difference of average speeds between Non-VSL, VSL, and IASLD under wet and icy conditions is lower than dry conditions.

Figures 17(a) and 17(b) illustrate the impacts of using Non-VSL, VSL, and IASLD approaches on average traffic flow in scenario of incident occurrence in the highway, under two conditions of dry and wet. For this experiment, we have created two lanes closure in the location of 6200 meters along the highway, which make an unpredictable bottleneck in this area. The results indicated that occurrence of incident had affected the traffic flow from the station 50 which is almost 3000 meters upstream of the incident location. The procedure of using variable speed limits in both of the VSL and IASLD approaches in comparison with Non-VSL approach resulted in amelioration of traffic flow volume in the 3000 meter distance prior to the incident location. From the other part, the consideration of multirestricted area as an integrated traffic controlling in IASLD has caused the dramatic increase of traffic flow volume (as it sensed in Non-VSL) to transform to the gradual increase of traffic volume, specifically in the 2500 meter distance prior to incident location. The improvement of traffic flow in IASLD rather than Non-VSL and VSL approaches for the distance of 2000 meter up to the distance of 6000 meters, respectively, has been 31.2% and 18.9% under the dry condition. Also this improvement under the wet condition has been 28.6% and 16.7%. The result shows that, in all the approaches, traffic volume pursues dramatic decrease after crossing the bottleneck (incident). We have disregarded to explain the evaluation of current approaches under the icy condition owing to approximative similarity of main impacts between this condition and two other conditions.

RETRACTED

Figures 18(a) and 18(b) clarify the reaction process of the IASLD and VSL to traffic congestion in the 240 seconds from the time of triggering the incident in aforementioned scenario of Figure 17(a) under the dry condition. In IASLD the speed buffering is applied 11.9 seconds after occurrence of incident; thus, the default speed of heavy congested condition is applied to the areas under authorization of stations 120, 110, 100, and 90. On the other hand, in VSL the first speed limit is applied 21 seconds after occurrence of incident to the area under authorization of station 120. Afterwards the subsequent speed limits are applied 112 and 148 seconds after occurrence of incident to the area under authorization of station 110. Lastly the station 100 applies the speed limit of 80 km/h in the time intervals of 228 seconds. Employment of immediate VANET-based incident detection beside consideration of speed buffering in SILID, contrary to depicted tardy procedure of traffic controlling in VSL, demonstrates the efficiency of integrated traffic controlling in IASLD which led to amelioration of traffic fluency.

For the performance evaluation of incident detection in IASLD, we have simulated the occurrence of incident (two lanes closure) in different traffic flows whereas the incident for each traffic flow is iterated three times at different locations of 3040, 6200, and 7250 meters along the highway. Then we have considered the detection evaluation from two distinct perspectives: (1) efficiency of detection procedure from the matter of time and accuracy; (2) considering the impacts of network's parameters alteration on the incident detection.  Table 6 depicts the values for average detection time—the average of time taken for detecting the incident warning message by RSU, from the initiation of incident; channel load—the load or share of the channel enforced by all the current messages propagating including the incident warning messages and advisory speed limit related messages; detection rate—specifying the ratio of the detected incidents using the VANET to all the incidents occurring in highway; false alarm rate—the ratio of the received false alarm messages, to all the received messages, which describe the performance of IASLD in different traffic volumes. The considered traffic volumes comprise 1000 vphpl to 1800 vphpl, describing the detected volume of the traffic by the closest loop detector prior to incident at the time of incident occurrence. The results demonstrate the preference of IASLD which had maximum detection time of 13.36 seconds; whereas the VSL requires great deal of time as a matter of congestion detection using the loop detector. Although the results showed the growth of channel load as a result of increasing the propagated advisory speed limit relating messages along the network, it did not have remarkable impact on latency of detection time. Moreover, the IASLD achieved the total average detection rate of 88% from all the applied incidents in simulation. The results showed that the probability of false alarm rate for incident detection was mainly affected by increasing the number of vehicles which had detected the emergency deceleration in the segments rather than the incident's segment due to growth of cluster's density nearby the incident.

RETRACTED

For evaluation of IASLD and VSL impacts on controlling the traffic congestions caused by growth in number of vehicles travelling in specific location of the highway, we have simulated the scenario of injecting the large number of vehicles to the entrance E23 prior to station 90 under the dry condition, whilst the average volume of the vehicles in station 90 has been 1430. Figures 19(a) and 20(a) illustrate, respectively, the IASLD and VSL impacts, on occupancy of highway segments which are affected by the traffic congestion. Thus, the alterations of occupancy parameters from the station 40 to station 90, in IASLD and VSL, from the initiation time of congestion detection until the end of simulation time are analyzed. In IASLD, the detection has been initiated (time 0) by perceiving the light congestion in station 90. Afterwards, there has been further detection of light congestion and moderate congestion in station 80 at the times 60 and 100, respectively. On the other hand, in VSL, by increasing the occupancy of vehicles more than the defined threshold in the station 90, and afterwards exceeding the volume, the new speed limits are applied, respectively, in times 0 and 140, to this station. The absence of integrated speed buffering along the consecutive segments in VSL caused the applying of new speed limits in stations 80, 70, and 60 to postpone to later time intervals at which the exceeding of occupancy and volume parameters is detected. Hence, every station has experienced a considerable rise in occupancy of vehicles before moderating the traffic flow. The comparison of IASLD and VSL in Figures 19(a) and 20(a) illuminates that IASLD had 8.1%, 7.9%, 20.8%, 28.9%, 26.8%, and 23.4 % improvements in reduction of occupancy, respectively, in stations 90, 80, 70, 60, and 50 rather than VSL after 320 seconds from first congestion detection. The represented contour maps in Figures 19(b) and 20(b) clarify the alterations of traffic congestions from the distance 2000 to 4500 meters of the highway during the 320 seconds from the detection of aforementioned congestion in IASLD and VSL approach, respectively. The depicted variation of density and occupancy in Figure 19(b) prominently indicates the influence of using gradual speed buffering directly on the traffic controlling of vehicles in IASLD, in the way that the density of traffic in stations 90, 80, 70,and 60 after 320 seconds from applying the speed limit policy is 34%, 18.1%, 19.2%, and 19.8% diminished, respectively. On the other side, Figure 20(b) manifests nonexistence of integrated traffic controlling, which correspondingly caused the VSL confronts with scattering of traffic congestion in prior stations by lapse of time.

Table 7 represent the average time of delivering the advisory speed limit to the vehicles in different volumes of traffic in IASLD approach. This amount is particularly the average of time intervals taken from initiation of sending the advisory speed limit packet until receiving the acknowledgement packet by the RSU. Moreover, Table 7 comprises the packet delivery ratio rate, which identifies the ratio of the number of advisory speed limit packets received to the receivers to the number of advisory speed limit packets sent by the RSU. The maximum average delivery latency obtained in volume of 2000 vphpl has been 1.68 seconds; hence, it denotes the efficiency of using VANET-based advisory speed limit delivered by considering this matter that initiations of “advisory speed limit propagation” procedure have been started prior to entering the vehicles to the segment where the advisory speed limit belongs to. On the other side, the obtained values for packet delivery ratio have been mainly above 80%. By increasing the volume of the traffic above 1600 vphpl, the growth of vehicles density in vicinity of RSU had led to reducing this value below the 80%, although it did not pass the threshold of 70% in traffic volume of 2000 vphpl as high density congestion.

RETRACTED

## 5. Conclusion

This study proposed IASLD as the VSL control strategy system which is able to determine advisory speed limits exclusively based on vehicle characteristics as well as traffic and weather conditions. The procedure of identifying the vehicles' characteristics is obtained by using series of image processing techniques. To reap benefits from a fast recognition times, probabilistic neural network (PNN) is chosen as a classifier. The traffic detection procedure in IASLD is composed from utilization of loop detectors and VANET technology. In addition, this approach takes advantage of VANET for providing the advisory speed limits of vehicles in successive segments of the highway. The presented simulations results demonstrate efficiency of IASLD in improving the traffic flow and occupancy of vehicles up to 28.9% in different traffic scenarios, where IASLD was applied in part of the 8 km network. The results also indicate that IASLD control strategy reduces the average travel times of the vehicles up to 9.3% in comparison with existing VSL approaches. Moreover, the results show that utilization of V2I communication in IASLD has evidently reduced the incident detection time up to 31.2% and 28.6 under dry and wet condition, respectively, where average detection rate of 88% was achieved from the entire applied incidents in the simulation. It is worth to note that the demonstrated efficiency of IASLD has been in condition that the driver compliance level was considered as an average value, which means that by increasing the level of driver compliancy the efficiency of IASLD will prominently improve.

## Figures and Tables

**Figure 1:** Fundamental layout of the VSL system.

**Figure 2:** Speed limit decision making structure in traditional VSLs.

**Figure 3:** Fundamental layout of the IASLD architecture.

**Figure 4:** Incident warning message structure.

**Figure 5:** Deployment of VANET-based incident detection along the highway.

**Figure 6:** Differentiation of stopping distances for vehicle equipped with ABS/EBD and unassisted vehicle.

**Figure 7:** License plate segmentation steps.

**Figure 8:** Vehicle classification identification after plate recognition.

RETRACTED

**Figure 9:** IASLD speed buffering in different traffic congestions scenarios.

**Figure 10:** IASLD advisory speed limit calculation procedure.

**Figure 11:** Beacon message structure.

**Figure 12:** Advisory speed limit requests message structure.

**Figure 13:** Advisory speed limit message structure.

**Figure 14:** Layout of the study section.

**Figure 15:** Impacts of Non-VSL, VSL, and IASLD on travel time in congestion-free scenario.

**Figure 16:** Impacts of Non-VSL, VSL, and IASLD on average volume of vehicles in congestion-free scenario.

**Figure 17:** (a) Impacts of Non-VSL, VSL, and IASLD on average volume of vehicles in incident occurrence scenario under the dry condition. (b) Impacts of Non-VSL, VSL, and IASLD on average volume of vehicles in incident occurrence scenario under the wet condition.

**Figure 18:** (a) Reaction time of VSL for applying the speed limits from the time of occurrence of the incident. (b) Reaction time of IASLD for applying the speed limits from the time of occurrence of the incident.

**Figure 19:** (a) Impact of IASLD on occupancy of highway segments which are affected by traffic congestion. (b) Alteration of traffic congestions in IASLD.

**Figure 20:** (a) Impact of VSL on occupancy of highway segments which are affected by traffic congestion. (b) Alteration of traffic congestions in VSL.

**Table 1:** List of acronyms.

Acronym	Definition
ABS	Anti-lock braking system
CCWS	Cooperative collision warning systems
CP	Crash potential
CRM	Coordinate ramp metering
DMS	Dynamic message sign
DSL	Differential speed limit
EBA	Electronic braking assist
EBD	Electronic brake force distribution
EDR	Event Data Recorder
GPS	Global Positioning System
IDS	Incident detection system
ITS	Intelligent transportation system
I2V	Infrastructure-to-vehicle
LP	License plate
LPR	License plate recognition
MANET	Mobile ad-hoc network
OBU	On-board unit
PNN	Probabilistic neural network
ROI	Region of Interest
RSU	Road side unit
RWIS	Road weather information system
SCW	Sliding concentric windows
SUMO	Simulation of urban mobility
SSD	Safe stopping distance
USL	Uniform speed limit
VANET	Vehicular ad-hoc network
VSL	Variable speed limit
V2I	Vehicle-to-Infrastructure
V2V	Vehicle-to-vehicle
WAVE	Wireless Access in Vehicular Environment

**Table 2:** The values of SSD-baselines according to the current Default speed of the highway area.

Default Speed limit		First SSD-baseline	Second SSD-baseline
1st and 2nd type	3rd type		
100 km/h	70 km/h	43.4 meters	42.6 meters
80 km/h	60 km/h	27.9 meters	31.2 meters
60 km/h	45 km/h	15.6 meters	17.7 meters
40 km/h	30 km/h	6.9 meters	7.8 meters

**Table 3:** The friction coefficient quantities for different vehicle classifications in different road conditions.

Road condition	Safety capability	Passenger Vehicles (first type)	Pickup and Van vehicles (second type)	Heavy vehicles (third type)
		Using first SSD-baseline		Using second SSD-baseline
Dry asphalt	Class B	0.9	0.75	0.45
	Class A	1.1	0.85	0.55

Wet asphalt	Class B	0.6	0.55	0.3
	Class A	0.7	0.6	0.35

Ice asphalt	Class B	0.15	0.12	0.1
	Class A	0.12	0.09	0.08

RETRACTED

**Table 4:** Plate processing and character recognition.

↓	Input: Image matrix A	
	crop	Utilizes of the coordinates in input (matrix A)
	name	Name the obtained image as *P*_1_

	resize	Make Standard size of 75 × 228 pixel from *P*_1_
	name	The obtained image as *P*_2_

	for	Each pixel in image *P*_2_{
	start	SCW method in *P*_2_
	parameters:	*X*_1_ = 2, *Y*_1_ = 5, *X*_2_ = 4, *Y*_2_ = 10, *T* = 0.7, *M* =
	and	standard deviation value; }
	name	The obtained image *P*_3_

	inverse	Image *P*_3_
	name	The obtained image as *P*_4_

	Run	Binary measurement in *P*_4_
	Retrieve	Objects which meet (orientation > 75 degree),
		(height > 32 pixels)
	name	The obtained image as *p*_5_

	Recognize	The bounding case of characters using standard deviation in *p*_5_

	run	Character segmentation in *p*_5_

	Count *c*,	Where *c*: NO. detected characters

	for	*a* = 1 : *c*,
	{convert	Character to 9 × 12 pixels

	create	Input vector
	Forward	Input vector to PNN and get decision }

**Table 5:** Simulation parameters summary.

Traffic and network related parameters	
Scenario dimension	8 km, 3 lanes, 1 direction
Maximum number of vehicles	400 vehicles for high traffic density
Number of vehicles for each type	75% passenger
	20% van
	5% heavy vehicle
Maximum vehicle speed	120 km/h
Assumed vehicle length	5 m, 6 m, 10 m
Regular deceleration	4.5 (m/s^2^)
Emergency deceleration	9 (m/s^2^)
Speed distribution	SpeedFactor 1
	SpeedDev 0.1
Minimum gap in high congested area	2 m
Intervehicle spacing	7–43 m
Driver imperfection value	0.5
Impatience value	0.8
Simulation time	400 s
Number of runs	15

Radio propagation model	Two-ray ground
Link/MAC layer protocol	IEEE 802.11p
Data rate	6 MB/s
Channel bandwidth	10 MHz
Channel frequency	5.9 GHz
Vehicles antenna gain	3 dBi
RSU antenna gain	10 dBi
Vehicle antenna height	1.5 m
RSU antenna height	9 m
Noise floor (thermal noise)	−104 dB_m_
Minimum contention window	15
Transmission power	
RSU	16.8 dB_m_
Vehicle	10.8 dB_m_
Receiver sensitivity	−91 dB_m_
Symbol duration	8 *μ*s
Clear channel assessment threshold	−65 dB_m_
SINR for preamble capture	5 dB
SINR for frame body capture	10 dB
Slot time	13 *μ*s
SIFS time	32 *μ*s
Preamble length	32 *μ*s
PLCP header length	8 *μ*s
Packet sizes	100, 200, 250 bytes
Beacon generation rate	5 Hz
Modulation	QPSK
Maximum communication range	300 m

RETRACTED

**Table 6:** Detection time, Channel load, Detection rate and False alarm rate of IASLD for different traffic volumes.

Volume (vphpl)	1000	1100	1200	1300	1400	1500	1600	1700	1800
Average detection time (s)	8.4	8.84	9.35	9.89	10.57	11.81	12.22	12.73	13.36
channel load (±0.1) (Mbps)	3.13	3.47	3.8	4.06	4.31	4.55	4.79	4.94	5.21
Detection rate	66% (2/3)	66% (2/3)	100% (3/3)	100% (3/3)	100% (3/3)	100% (3/3)	66% (2/3)	100% (3/3)	100% (3/3)
False alarm rate	0.2%	2.3%	5.3%	8.8%	11.1%	12.9%	15.4%	17%	18.6%

**Table 7:** Average advisory speed limit delivery latency of IASLD in different traffic volumes.

Volume (vphpl)	Average Advisor speed delivery latency	Packet Delivery ratio
100	N/A	N/A
200	216.1	0.987
300	218.3	0.964
400	256	0.953
500	281	0.951
600	319.4	0.938
700	377.2	0.92
800	441.6	0.904
900	490.2	0.891
1000	562.3	0.889
1100	649	0.867
1200	731.8	0.858
1300	761.1	0.841
1400	834.8	0.816
1500	923.4	0.801
1600	1017.9	0.792
1700	1262.7	0.774
1800	1484.2	0.753
1900	1551.5	0.728
2000	1689.1	0.703
